# Design and Implementation of Interactive Platform for Operation and Maintenance of Multimedia Information System Based on Artificial Intelligence and Big Data

**DOI:** 10.1155/2022/4620930

**Published:** 2022-05-04

**Authors:** Xin Yan, Junhui Yan

**Affiliations:** ^1^School of Management, Shanghai University, Baoshan, Shanghai 200444, China; ^2^Maths & Information Technology School, Yuncheng University, Yuncheng, Shanxi 044000, China

## Abstract

In order to cope with the challenges that operators face after the impact of diversified social channels in the field of interactive services, we actively build a new generation of intelligent interactive systems based on artificial intelligence technology, a semantic understanding, and intention recognition, covering rich media content, omnichannel coverage, high-frequency knowledge updates, consistent service response, high-quality, and low-cost intelligent interactive solutions is proposed. The solution provides overall business modeling for scenario design and a scenario-based knowledge expression system, with the function of fragmented knowledge processing. With complete text and voice information, combined with pictures, text, audio, video, and other multimedia, we intelligently interact with users, allowing users to obtain required information and solve problems in a pleasant and relaxing interaction. Therefore, the research and exploration of the intelligent interactive system architecture based on artificial intelligence is a useful practice and strong support for operators to redefine the connotation and elements of “smart service” in the process of building “smart operation.” Through repeated tests, it can be seen that the language similarity has reached 0.75549, which is very close to 1.0000. It can be seen that the design of this platform has been successful.

## 1. Introduction

Since the 21st century, with the rapid development of computers and networks, artificial intelligence has become the most popular technology term today. The development of artificial intelligence affects the development of all walks of life. The development of robotics, autonomous driving technology, image recognition, and other technologies indicates that artificial intelligence is getting more and more attention from people, and its development has great potential. Big data plays a vital role in the development of artificial intelligence. Through the relationship between artificial intelligence and big data, starting from their development status, this article describes in detail the future development trend of artificial intelligence in the big data environment. The robot operating system ROS is easy to use [1]. After determining the functional modules that the human-machine voice interaction system should have, we use the topics and services provided by ROS to realize the communication between related modules in the system and define the information format during communication. ROS originated from the cooperation between the STAIR project of the Stanford University Artificial Intelligence Laboratory in 2007 and the personal robot project of the robotics company Willow Garage. After 2008, Willow Garage promoted its development. ROS is an open-source meta-operating system suitable for robots. It provides the functions that the operating system should have, including hardware abstraction, low-level device control, realization of common functions, interprocess information transmission, and software package management. In addition, it also provides the tools and libraries needed to compile, write, and execute programs across multiple computers [2]. ROS is similar to Player, YARP, Orocos, CARMEN, Orca, MOOS, and Microsoft Robotics Studio robot frameworks in some respects. The “blueprint” of the ROS runtime is a loosely coupled point-to-point process network based on the ROS communication infrastructure. ROS has several different communication methods, including a service mechanism based on synchronous remote procedure call protocol (Remote Procedure Call Protocol, RPC) communication, a topic mechanism based on asynchronous streaming media data, and a parameter server for data storage [3].  Figure 1 shows the flow chart of the intelligent interactive system management platform. Big data uses the increasingly mature cloud computing technology to obtain valuable information from the vast ocean of Internet information for information induction, retrieval, and integration, providing a software foundation for Internet information processing. Both require the participation of artificial intelligence, which is a commercial application after the order of the Internet information system. That is the real outlet for cloud computing and big data.

## 2. Literature Review

Tekerek A. and others said that the arrival of the era of intelligence and big data, and the social impact brought about by the industrial revolution in history, have inherent laws that are similar in appearance and similar in quality to the contradictions and mutual influences between productivity and production relations [4]. Ha T. and others stated that the era of intelligence and big data seems to have provided greater “convenience” for “distrust, disorder, and monopoly,” and at the same time put forward higher requirements for “trust, order, and sharing [5].” Kyivska K. and others said that in the past 20 years, with the rapid development of artificial intelligence technology, especially the intelligence and big data information economy characterized by “Internet +,” it has almost reshaped the production and operation models of enterprises and people's way of life has had a significant impact on the transformation of the paradigm of human “technology-economy-society” and the progress of social civilization [6]. Ongena et al. said that with the widespread application of computer technology, the continuous increase in data accumulation, and the continuous innovation and enhancement of algorithms and computing power, the current society has entered the era of intelligence [7]. Through research, Bhargava et al. have obtained the development of the “four major catalysts” of massively parallel computing, big data, deep learning algorithms, and smart chips, as well as the reduction of computing costs, which has enabled artificial intelligence technology to advance by leaps and bounds [8]. Fanea and others said that artificial intelligence has become the most exciting and most anticipated technology of this era, and it will become the focus of the development of the IT industry in the next 10 years and beyond [9]. Naghizade et al. found through investigations that the current operators are also facing the impact of the mobile Internet. Diversified service requirements, diversified service scenarios, and fragmented social service models are all impacting the traditions of operators from all angles. *Service interaction mode* [10]. Zhang et al. said that the response speed and service satisfaction of interactive services force operators to innovate the service interaction model. The high-frequency requirements for service personnel knowledge update and training cost control have promoted the traditional interactive service model to the network. Development in the direction of automation, automation, and intelligence, through rich media and multichannels to achieve intelligent interaction with users, and effectively reducing service costs, improving service quality, and increasing user perception are the current urgent needs, which have been listed by operators as building the key issue of “smart operation” [11]. Elayyan and others said that with the development of artificial intelligence, the research of robots has also made great progress. Robots of various forms and functions have appeared one after another, and some robots have even entered people's homes and become members of the family [12]. Batarseh and others stated that the most important way for humans to interact with robots is through voice, which is more direct and convenient than other methods such as buttons, touch screens, and remote controls. Therefore, a human-machine with good performance is designed in the development of robots. The voice interaction system is very important. The intelligence of the robot must first be manifested in the smooth human-machine voice interaction function. The human-machine voice interaction system has become the most basic functional design requirement [13].

This paper combined with the requirements of information technology service-related standards and specifications, as well as the operation and maintenance project implementation experience and the key generic technology for information system operation and maintenance, provide system support for information system operation and maintenance specification, realize the information system operation and maintenance support system software industrialization and operational service interactive development pattern, drive the market demand of information system operational service, and promote the rapid formation and healthy development of operation and maintenance service industry chain.

## 3. Method

### 3.1. Use Bayesian Algorithm to Achieve Text Classification

Big data has now been summarized as having the characteristics of 4v: volume, velocity, variety, and value. The total data growth is shown in Figure 2.

Big data is a brand-new business model, life philosophy, and ideology developed on the basis of multiple data and cross-domain associations. This new approach to tools will have a huge disruptive impact on all aspects of our society. This is summarized on the basis of the characteristics of big data. With the continuous development of big data, when it reaches the advanced stage, it will generate new value and bring a qualitative leap to all aspects of society such as enterprises and schools [14]. There are many classic classification methods in machine learning, such as decision tree algorithms, support vector machines, Bayesian classification algorithms, artificial neural networks, and k-nearest neighbors. To process the text recognized by the speech recognition function, and to deal with the text classification problem, the naive Bayes classifier is one of the most effective algorithms. There are three reasons why Bayesian algorithm is often used to achieve text classification. First, the Bayesian algorithm is simple; second, it is easy to get the probability value required to train the Bayesian classifier based on the training text; third, naive Bayes classifier is comparable to other algorithms in most cases, and in some cases even better than other algorithms. The classification problem is the process of finding the best hypothesis from the hypothesis space given the training data. For sentence text Q, we can denote it as 〈*a*_1_, *a*_2_,…, *a*_*n*_〉 after word segmentation, where *a*_*i*_(1 ≤ *i* ≤ *n*) represents the word in sentence Q [15]. The classification of Q in this article is to divide it into a certain category of daily life frequently asked question and answer library, professional field frequently asked question and answer library, real-time question library, or control instruction library, that is, to deal with the following questions:

(1) $$\begin{array}{c} v_{\text{MAP}}=\underset{v_{j}\in V}{\arg\;\max}P\left(v_{j}|a_{1},a_{2},\ldots ,a_{n}\right), \end{array}$$

where *v*_MAP_ represents the maximum posterior value; V represents the category set of the library composed of the daily FAQ library, the professional field FAQ library, the real-time question library, and the control instruction library; and the *v*_*j*_ is the category that Q can be divided into [16]. Using Bayesian formula, formula (1) can be rewritten as

(2) v=MAParg maxvj∈VPa1,a2,…,an|vjPvjPa1,a2,…,an=arg maxvj∈VPa1,a2,…,an|vjPvj,

where *P*(*v*_*j*_) represents the probability of each target value *v*_*j*_ and *P*(*a*_1_, *a*_2_,…, *a*_*n*_*|v*_*j*_) represents the probability of 5 under the condition of the target value *v*_*j*_. We can get *P*(*v*_*j*_) by counting the number of frequently asked questions in daily life, frequently asked questions in professional fields, real-time question banks, or control instruction banks. But to get the value of *P*(*a*_1_, *a*_2_,…, *a*_*n*_*|v*_*j*_), a large training data set is required. In order to reduce the amount of calculation, it can be assumed that the words *a*_*i*_(1 ≤ *i* ≤ *n*) in the sentence are independent of each other, which reduces the problem to a naive Bayes classification problem. The corresponding formula (2) can be simplified as follows:

(3) $$\begin{array}{c} v_{NB}=\underset{v_{j}\in V}{\arg\;\max}P\left(a_{1},a_{2},\ldots ,a_{n}|v_{j}\right)P\left(v_{j}\right)\\ =\underset{v_{j}\in V}{\arg\;\max}P\left(v_{j}\right)\prod_{i}P\left(a_{i}|v_{j}\right), \end{array}$$

where *v*_*NB*_ represents the target value output by the naive Bayes classifier, *P*(*v*_*j*_) represents the probability of each target value *v*_*j*_, and *P*(*a*_*i*_*|v*_*j*_) represents the probability of word *a*_*i*_(1 ≤ *i* ≤ *n*) under the condition of the target value *v*_*j*_. To use the naive Bayes classifier to deal with the sentence text classification problem, at this time, we only need to estimate *P*(*v*_*j*_) and *P*(*a*_*i*_*|v*_*j*_) from the training data [17].

### 3.2. Human-Machine Voice Interaction System Based on ROS

The execution process of the designed ROS-based human-machine voice interaction system is shown in Figure 3.

The main functions in the human-machine voice interaction process are described in detail below.

#### 3.2.1. Voice Information Collection

The voice information is collected through the external microphone of the robot, and the collected voice information is stored as an audio file. The quality of user voice information collected in a noisy environment will be disturbed by noise. In addition, it is impossible to know in advance when the user will speak to the robot, whether he is talking to the robot, and the duration of the speech. Therefore, the problems of noise interference, when to collect the user's voice information, and the collection time must be solved first [18]. These problems can be solved by voice activity detection (voice activity detection, VAD) technology. Voice endpoint detection technology is a basic link in speech recognition and speech processing, and it is also a popular field of speech recognition research. Its main purpose is to distinguish speech and nonspeech from the input speech. The main functions are automatic interruption, removal of silent components in the voice, obtaining effective voice in the input voice, and removing noise to enhance the voice. The open-source project pyVAD on GitHub is used to implement endpoint detection on the voice data read in real time.

#### 3.2.2. Voice Recognition Node

The voice recognition node is responsible for recognizing the collected voice information as text information. This article uses the REST API provided by Baidu voice to implement speech recognition. The speech recognition REST API provides developers with a universal HTTP interface that supports the POST method [19]. Based on this interface, developers can easily implement speech recognition functions. The API supports the recognition of the entire recording file; that is, the user needs to upload the entire voice, but the original voice file must conform to the specified format.

#### 3.2.3. Speech Synthesis Node

The speech synthesis node is responsible for synthesizing the requested information into audio. The speech synthesis is realized by using the REST API provided by Baidu voice. Speech synthesis REST API supports the synthesis of a paragraph of text, but the text must be encoded in UTF-8, and the text length must be less than 1024 bytes [20]. Currently, the interface supports both POST and GET methods.

#### 3.2.4. Semantic Analysis Node

The semantic analysis node has the function of understanding the request information received from the speech recognition node to determine what operation the robot should perform. The semantic analysis node must not only provide services to the speech recognition node but also must be able to request services provided by other nodes or publish information on specific topics [21].

#### 3.2.5. Real-Time Information Acquisition Node

Through real-time information acquisition nodes, real-time changing information content, such as time, date, weather, and news, can be obtained. Nodes that provide time and date information access services, and nodes that provide weather access services in major cities are now implemented [22].

#### 3.2.6. Robot Control Function Node

The robot control function nodes include nodes that control the robot to walk, avoid obstacles, and reach designated positions. These nodes need to be developed separately. On the PC side, the robot's walking function is tested and controlled by the turtlesim software package officially provided by ROS, and the function of playing music through voice control is also realized. On the built robot platform, the Python program that controls the movement of the motor is written through the GPIO port to realize the control of the robot [23].

## 4. Results and Analysis

Through analysis, the steps to classify sentence text Q are as follows:

**Step 1 .**

Collect and connect the question item in the FAQ database of daily life as a document and record it as category 1. Collect and connect the question item in the FAQ database of each professional field as a document and record it as category 2 (for convenience Explain that it is assumed that there is only one frequently asked question library in the professional field); the question item in the collection and connection real-time question library is a document, which is recorded as category 3; the question item in the collection and connection control instruction library is a document, and is recorded as category 4 [24].

**Step 2 .**

Combine all categories of documents into a document, use Chinese word segmentation method to segment the Document, collect all the words in the Document, and form a collection Vocabulary. All categories form a set *V*, that is, *V* = {category 1, category 2, category 3, category 4}.

**Step 3 .**

For each target value *v*_*j*_ in *V*, calculate the probability term *P*(*v*_*j*_):

(4) $$\begin{array}{c} P\left(v_{j}\right)=\frac{\left|{\text{docs}}_{j}\right|}{\left|\text{Document}\right|}, \end{array}$$

where docs_*j*_ is the subset of documents whose target value is in Document, |docs_*j*_| is the number of elements it has, and |Document| is the total number of category libraries that Document has [25].

**Step 4 .**

For each target value *v*_*j*_ in *V*, connect all members in docs_*j*_ to build a document Text_*j*_, use Chinese word segmentation method to segment *Text*_*j*_, and count the number *n* of different words in Text_*j*_.

**Step 5 .**

For each word *a*_*i*_ in Vocabulary, calculate the probability term *P*(*a*_*i*_*|v*_*j*_):

(5) $$\begin{array}{c} P\left(a_{i}|v_{j}\right)=\frac{n_{k}+1}{n+\left|\text{Vocabulary}\right|}, \end{array}$$

where *n*_*k*_ is the number of occurrences of word *a*_*i*_ in Text_*j*_, and |Vocabulary| is the total number of words that Vocabulary has [26].

**Step 6 .**

Use the Chinese word segmentation method to segment the sentence *Q* to get 〈*a*_1_, *a*_2_,…, *a*_*n*_〉, where *a*_*i*_ represents the word that appears at the i-th position in *Q*.

**Step 7 .**

Get the category *v*_*NB*_ to which *Q* belongs

(6) $$\begin{array}{c} v_{NB}=\underset{v_{j}\in V}{\arg\;\max}P\left(v_{j}\right)\prod_{i\in \text{positions}}P\left(a_{i}|v_{j}\right), \end{array}$$

where positions are the position where all words appear in *Q*. Any words that appear in *Q* but not in the documents in the training set will be simply ignored [7].

In order to verify the performance of the proposed ROS-based human-machine voice interaction system, experiments were carried out on the PC terminal and the robot platform built in the laboratory to test the human-machine voice question and answer function and the robot control function [27]. PC environment: Ubuntu 12.04, 32-bit operating system, the processor is Pentium(R) Dual-Core CPU E6500 @2.93 GHz 2. Install the robot operating system ROS on the Ubuntu system and choose Hydro as the ROS version. Sound collection device: USB microphone. Audio playback equipment: USB stereo. The robot platform is built on the HCR (Home Care Robot) omnidirectional wheel development platform. The central processor of the robot platform uses Raspberry Pi 2B, and the system installed on the Raspberry Pi is Raspbian wheezy. Install ROS on the Raspberry Pi, and the ROS version is Hydro. The GPIO port is used to control the rotation of the motor to make the robot walk. The motor drive module adopts SKU: DRI0018. Use a USB microphone to collect voice information and use a USB speaker to play audio.

As can be seen from Figure 4, after data smoothing, the obtained sample data are sorted from small to large. In order to ensure that all data are generated under nonabnormal conditions, the smallest and largest numbers need to be eliminated. The obtained data are as follows: [24, 34, 38, 39, 39, 39, 41, 41, 51, 53, 54, 56, 63, 63, 66, 67, 69, 73, 78, 79, 79, 79, 81, 87, 89, 91, 94 ,99, 102, 103]. Determine the range of 5 intervals, 103/5 = 21, namely, [0∼21], [21∼42], [42∼63], [63∼84], and [84∼105]. Distribute the remaining 28 numbers after removing the abnormalities into these 5 intervals (interval minimum value ≤ *N* < interval maximum value). Interval 1 = ; Interval 2 = [34, 38, 39, 39, 39, 41, 41]; Interval 3 = [51, 53, 54, 56]; Interval 4 = [63, 63, 66, 67, 69, 73, 78, 79, 79, 79, 81]; interval 5 = [87, 89, 91, 94, 99, 102]. After interval allocation, it can be seen that the number of data in interval 4 is the largest. Therefore, the data in interval 4 and the upper and lower adjacent intervals 3 and 5 are taken. If there are no data in the upper and lower adjacent intervals, it is not necessary to take them. 21 data can be obtained [28].

The daily life frequently asked question and answer library established during the experiment contains 15 question and answer pairs, the library frequently asked question and answer library contains 50 question and answer pairs, the real-time question library contains 19 questions, and the control instruction library contains 30 instructions. The similarity value is a unitless real number in the interval of [0,1]. The closer the value is to 1, the more similar the meaning of the two sentences, and vice versa. Regarding the calculation of similarity, several existing basic methods are all based on vectors. In fact, it is to calculate the distance between two vectors. The closer the distance is, the greater the similarity. In the recommended scenario, in the two-dimensional matrix of user-item preferences, we can use a user's preference for all items as a vector to calculate the similarity between users, or use all users' preferences for an item as a vector A vector to calculate the similarity between items.

In order to test the performance of the similarity calculation method, three question items from the daily FAQ database were selected as “question sentences,” and the similarity values between these three questions and each question item in the daily FAQ database were calculated.  Table 1 lists the first three largest similarity values obtained in each calculation. The similarity value of each question in the table with itself is 1.00000.

Table 2 shows the similarity values between the three question sentences and the three question items in the library frequently asked questions and answers library.

Table 3 shows the similarity values between the question sentences expressing the same meaning and the question items in the library frequently asked questions. From the results in Table 3, it can be seen that for the same subject matter, if different questioning methods are used, it can also be well matched to the question item in the library. The adopted sentence similarity calculation method has strong adaptability to a variety of questioning methods.

Three question items are selected from the real-time question database as question sentences, and the similarity values between these three question sentences and each question item in the real-time question database are calculated, respectively.  Table 4 lists the first three largest similarity values obtained in each calculation. The similarity value of each question in the table with itself is 1.00000.

The question “What's the time now?” is the same as the question item “What time is it now” and “Do you know what time it is?” The question “Do you know today's date?” expresses the semantic content of “date query,” and the question item “What is today's date?” The similarity value is 0.62517. The question item “Tell me today's date?” is the same as the semantic content of the question sentence, but the similarity value between the two is relatively small. It can also be seen from this that only relying on the Chinese knowledge dictionary and the number of identical words contained in the two sentences to measure the similarity between sentences cannot achieve very good performance, and the similarity calculation method can be further optimized.

## 5. Conclusion

From Table 1 above, it can be seen that the question “What is your name?” and the question item “What your name is it?” express the same semantic content, and the similarity value calculated by the experiment is 0.74825. And “Do you know what my name is?” is different from the semantic content of the question sentence, “Do you know what my name is?” is the user asking the robot his name, and “What is your name?” the user asking the name of the robot. Although the two sentences are intended to obtain names, the objects of the names to be obtained are different, so the calculated similarity value is relatively small. The question “What do you do?” and the question item “What can you do?” express the same semantic content, but the calculated similarity value is 0.48597, which shows that the sentence similarity calculation method adopted has room for improvement. The question “Do you know me?” and the question “Do you know what my name is?” are both the user asking the robot for his name. The calculated similarity value is 0.75549, which is very close to 1.00000.

The combination of interactive systems and artificial intelligence has greatly improved the accuracy and friendliness of interactive services. But at the same time, higher requirements are put forward for knowledge processing and learning, semantic intent recognition, interactive scenarios, and multiple channels. From the perspective of “achievable and deployable,” the construction of an intelligent interactive system architecture based on artificial intelligence provides functional design and optimized solutions to current problems and challenges, so as to further make interactive services more intelligent and rich, humanized, and convenient. It lays the foundation for the subsequent formation of an intelligent interactive product system that can be promoted, replicated, and reduced in cost and increased efficiency. The experimental results show that the design achieves small positioning error; improves the system accuracy; greatly facilitates the installation, debugging, and maintenance of the positioning network; and reduces the labor cost of the network layout.

The implementation of the information operation and maintenance comprehensive supervision system has undergone a lot of preparations, but due to the large number and variety of information system equipment involved in the monitoring of the system, the realization of some functions in the implementation process is not satisfactory, and the system is still in application. There are areas that need further improvement, and its shortcomings are summarized as follows:

1. The host, network, middleware, database, information security, and terminal equipment in the implementation of the information operation and maintenance comprehensive supervision system all involve alarm content. Due to the limited display interface, it cannot be displayed on the same interface. The real-time monitoring of information system monitoring personnel monitoring work increases the workload.
2. Since there are many types of information system software and hardware that enterprises need to monitor, the display center needs to display network, application system, and performance data on multiple interfaces, which brings a lot to the daily monitoring work of operation and maintenance monitoring personnel of greater pressure.

## Figures and Tables

**Figure 1:** Flow chart of the intelligent interactive system management platform.

**Figure 2:** Growth graph of total data.

**Figure 3:** Human-machine voice interaction system execution process.

**Figure 4:** Data smoothing calculation data diagram.

**Table 1:** Examples of the calculation results of sentence similarity in the FAQ database of daily life.

Question	The question item in the frequently asked questions and answers library of daily life	Similarity value
What's your name?	What's your name?	1.00000
	What's your name?	0.74825
	Do you know what my name is?	0.68549

What do you do?	What do you do?	1.00000
	What can you do?	0.48597
	What's your name?	0.34859

Do you know me?	Do you know me?	1.00000
	Do you know what my name is?	0.75549
	Do you know who I am?	0.58165

**Table 2:** Example 1 of sentence similarity calculation results in the library frequently asked questions and answers database.

Question	The question item in the library frequently asked questions and answers library	Similarity value
*What if the library does not have the books and periodicals I need?*	What if the library does not have the books and periodicals I need?	1.00000
	Can I borrow books and periodicals in the reading room? How long can I borrow?	0.32812
	How to recommend a good book to the library for purchase?	0.16829

*Do I need to submit a dissertation?*	Do I need to submit a dissertation?	1.00000
	How to submit a paper dissertation?	0.58294
	How to check the electronic version of the dissertation review results?	0.35059

*How to apply for one pass?*	How to apply for one pass?	1.00000
	About the one pass card	0.45027
	The all-in-one card is reported to be lost or reissued	0.29153

**Table 3:** Example 2 of sentence similarity calculation results in the library frequently asked questions and answers database.

Question	The question item in the library frequently asked questions and answers library	Similarity value
*What should I do if the library does not have the book I want to borrow?*	What if the library does not have the books and periodicals I need?	0.63967
	My library personal information	0.54045
	Why cannot the book that has just been returned be lent out again by the person returning the book?	0.32829

*What should I do if I do not find the book I need in the library?*	What if the library does not have the books and periodicals I need?	0.72000
	My library personal information	0.51294
	How can I collect items lost in the library?	0.42059

*What should I do if the journal I want to borrow is not in the library?*	What if the library does not have the books and periodicals I need?	0.65000
	My library personal information	0.49027
	What is my library account password?	0.47153

**Table 4:** Examples of sentence similarity calculation results under the real-time question bank.

Question	The question item in the frequently asked questions and answers library of daily life	Similarity value
*What time is it now?*	What time is it now?	1.00000
	What time is it now?	0.88205
	Do you know what time it is now?	0.82591

*Do you know what's the date today?*	Do you know what's the date today?	1.00000
	What's the date today?	0.62517
	Tell me today's date?	0.28405

*How's the weather today?*	How is the weather today?	1.00000
	How is the weather tomorrow?	0.75755
	Tell me how is the weather today?	0.74058

## Data Availability

The data used to support the findings of this study are available from the corresponding author upon request.
